The article "Head CT Image Segmentation and Three-Dimensional Reconstruction Technology Based on Human Anatomy" was published in 2022. Journal: Comput Intell Neurosci.

# Head CT Image Segmentation and Three-Dimensional Reconstruction Technology Based on Human Anatomy

**DOI:** 10.1155/2022/7091476

**Published:** 2022-06-16

**Authors:** Zhenyu Wu, Lin Wang, Yifei Li, Shuhui Dai, Dongliang Zhang

**Affiliations:** ^1^Department of Anatomy, Histology and Embryology and K.K. Leung Brain Research Centre, The Fourth Military Medical University, Xi'an 710032, China; ^2^Department of Neurosurgery, Xijing Hospital, Fourth Military Medical University, Xi'an 710032, China; ^3^Department of Burns and Cutaneous Surgery, Xijing Hospital, The Fourth Military Medical University, Xi'an 710032, China

## Abstract

With the continuous development of computer science and technology, the level of medical image processing and analysis technology has been significantly improved. In order to further optimize the medical imaging technology and provide assistance for medical diagnosis and treatment, this study will explore the head CT image segmentation technology and three-dimensional reconstruction technology based on human anatomy, using two morphological operation methods of image expansion and image corrosion, as well as the triangulation method based on surface contour, Optimize CT image segmentation technology and three-dimensional reconstruction technology. The results show that the CT image segmentation technology based on human anatomy can obtain the more essential morphology and features of the target image, and significantly improve the image quality. The size of the threshold can have a certain impact on the 3D reconstruction effect and reconstruction time to a certain extent. The larger the threshold, the shorter the reconstruction time, but the worse the 3D reconstruction effect. This shows that the target image after fitting has a good reconstruction effect, but the threshold level should be kept at a low level. The head CT image segmentation technology and three-dimensional reconstruction technology based on human anatomy have good application effects and can be popularized and applied in clinical diagnosis and treatment.

## 1. Introduction

In the process of the continuous development of medical technology, the application scope of human anatomy has been significantly expanded. Applying it to the image segmentation of head computed tomography (CT) can improve the effect of medical image segmentation to a certain extent [1]. The application of medical impact processing and analysis in clinical medicine is extremely critical and has attracted more and more attention. In order to improve the accuracy and reliability of medical diagnosis, it is imperative to explore and optimize medical image segmentation and processing technology and three-dimensional reconstruction technology [2]. CT image segmentation and processing technology plays an important role in the diagnosis and detection of head tumors. It can effectively realize image segmentation and processing when the boundary between normal head and diseased soft tissue is poor [3]. Three-dimensional reconstruction technology is a visualization means of scientific calculation, which can effectively analyze the calculation results of computer data and understand the changes of data in the calculation process under the action of computer graphics and image processing technology [4]. In view of this, this study will make a detailed exploration on the head CT image segmentation and three-dimensional reconstruction technology based on human anatomy, in order to improve the effectiveness of image segmentation and processing technology and three-dimensional reconstruction technology and promote the sustainable development of medical image processing technology.

This study mainly discusses the mechanism and application effect of head CT image segmentation technology and three-dimensional reconstruction technology in the context of human anatomy. Morphological operation is mainly used to explore the segmentation technology of head CT image. Morphological operation can effectively repair the area of the target CT image. Under the action of image expansion and image corrosion, head CT image can be well segmented. In addition, the surface rendering method in three-dimensional reconstruction technology is also analyzed in detail. This method is a triangulation method based on surface contour, which can use the small plane with the shape of triangle or polygon to place it in the boundary contour line as a filler to form a complete and smooth object surface. The combination of the two research methods provides strong support for exploring the application effect of head CT image segmentation and three-dimensional reconstruction technology.

In this study, the most innovative point is that in morphological operation, two operation methods of image expansion and image corrosion are used at the same time, which can effectively deal with the diversified problems in image segmentation. This innovative method can separate two connected objects on the basis of filling the hole after image segmentation so that the target image is not negatively affected by its own internal segmentation or external object adhesion, which can significantly improve the technical level of CT image segmentation and obtain more objective and accurate image segmentation results. Moreover, the research also innovatively makes a comprehensive comparative analysis of the threshold, three-dimensional reconstruction effect, and reconstruction time, which makes the application process of three-dimensional reconstruction technology not only blindly improve the threshold level but also comprehensively consider the impact of reconstruction efficiency and reconstruction effect.

The main structure of the paper is divided into four parts. The core content of the second part is to explore the research progress of many experts and scholars at home and abroad in CT image segmentation technology and three-dimensional reconstruction technology and briefly discuss its research means and research results. The third part mainly probes into the action mechanism of the two core technologies in this research, including the binarization processing of head CT image segmentation technology, the repair and merging of image regions, the construction of the contour model, the triangulation surface drawing method of three-dimensional reconstruction technology, and the simplification processing method of the triangular mesh. The fourth part focuses on the analysis of the application effect of head CT image segmentation technology and three-dimensional reconstruction technology. The fifth part mainly expounds all the research work and research results, summarizes the disadvantages and deficiencies, and looks forward to the future research direction.

## 2. Related Work

In recent years, medical diagnosis and treatment methods have been fully developed in the process of clinical application of medical imaging technology. However, in order to prevent the distortion of lesion target location and improve the effectiveness of medical diagnosis and treatment, the research on medical image processing technology at home and abroad has been continuously promoted and gradually deepened. Mason et al. believe that the current treatment workflow based on cone beam computed tomography (CBCT) is easily limited by the contrast difference of soft tissue. Therefore, ultrasonic fusion CBCT is used to compare and analyze the consistency and confidence of images. The accuracy of image segmentation and location is successfully improved [5]. Aiming at the problem of great difficulty and variability in liver segmentation, researchers such as Mourya et al. used CT image segmentation technology to eliminate the lack of clear edge of the liver boundary, significantly estimated the area of liver tumor, and carried out accurate automatic segmentation [6]. Selvaraj et al. used CT for image scanning and quantitative processing to solve the problem of Covid-19 area contour description and successfully realized the effective segmentation of Covid-19 infection severity [7]. Zeng et al. found that it is difficult to realize the automatic segmentation of head image from ultrasonic image and head circumference biometrics. By using DAG v-net deep learning model, CT technology was used to segment fetal ultrasonic image effectively [8]. Eckl et al. believe that image-guided radiotherapy can benefit from the implementation of radiotherapy technology. They have completed the construction and training of body part-specific model by evaluating the conversion algorithm from cone beam computed tomography to synthetic CT based on cyclic generation countermeasure network. Finally, CT images with high quality were generated [9]. Tappeiner et al. found that in the process of radiotherapy for head and neck cancer, the focus is to accurately depict the organs with risk in the image. The study used the method of deep learning combined with CT to effectively train the data set and successfully obtained the segmented image with high accuracy [10].

Yamamoto et al. conducted in-depth research on osteoclasts, used continuous section scanning electron microscope technology and three-dimensional reconstruction technology to reconstruct osteoclasts, and successfully found the unique three-dimensional shape of Golgi [11]. Yushan et al. analyzed rare congenital malformations and their related characteristics, achieved surgical reduction by using image technologies such as three-dimensional reconstruction, and finally achieved a better effect of surgical intervention [12]. In order to improve the accuracy and reliability of 3D reconstruction, Xie et al. applied the multiview photometric stereo fusion algorithm to 3D reconstruction technology and verified it through multiple iterations. Finally, the 3D reconstruction results with higher precision surface normals and better quality were successfully obtained [13]. Wang et al. believed that the two-dimensional image has the characteristics of fast but simple, so they applied the mobile robot vision technology to it, improved it, proposed the three-dimensional reconstruction technology, and verified the efficiency and accuracy of the three-dimensional reconstruction technology through simulation analysis [14]. Ruiz et al. proposed a nonrigid object 3D reconstruction algorithm using depth camera, which can dynamically construct the dense 3D model of the target object, improve the accuracy of 3D reconstruction, and can be applied to many fields such as medicine, agriculture, and human-computer interaction [15]. Jani et al. found that the application of three-dimensional technology in the reconstruction and description of human bone fragments is less. By analyzing the application of three-dimensional model in forensic cases, the accuracy of three-dimensional reconstruction model is improved from the perspective of anatomical features and digital analysis, and the optimization of three-dimensional reconstruction technology is realized [16].

By analyzing the research results of many scholars at home and abroad in CT image segmentation and three-dimensional reconstruction technology, it can be found that these two technologies have made great progress and have a wide range of applications, especially medical diagnosis and treatment. CT image segmentation technology and three-dimensional reconstruction technology can reflect a good application effect in medical diagnosis and more intuitively and accurately present the image information of the focus, which is convenient for later clinical treatment intervention. In view of this, this study takes human anatomy as the basic basis to deeply explore CT image segmentation technology and three-dimensional reconstruction technology in order to improve the accuracy of medical image segmentation and three-dimensional reconstruction.

## 3. Research on CT Image Segmentation Technology and Three-Dimensional Reconstruction Technology

### 3.1. Patching and Merging of Image Regions and Construction of Contour Model

In the actual process of computed tomography, X-rays are projected and scanned at different angles only in specific faults, and then, the corresponding projection and scanning results are handed over to the computer for further processing so as to obtain the two-dimensional projection distribution results of specific faults in the object to be measured. In the context of human anatomy, there are some differences between various human tissues and other objects. Taking the head as an example, when forming the CT image of the head, the X-ray absorption of the head tissue is different, so the CT image segmentation technology segments a section of the head tissue, and the small cube obtained after segmentation is voxel. When X-ray passes through the head, the density or gray level in each single voxel is measured as a pixel, that is, the basic unit in CT image. Before applying CT image segmentation technology, it is necessary to binarize the image. Usually, threshold segmentation based on image histogram is adopted as shown in Figure 1.

Figure 1(a) is a single-threshold histogram. Its segmentation principle is to use a threshold *T* to classify the gray level of the target image, determine the pixels whose gray value is in the same gray range as the segmented image from the same target, and finally realize accurate segmentation of the target image. The segmentation principle of the multithreshold histogram shown in Figure 2(a) is basically consistent with that of the single-threshold histogram. The difference is that more than one threshold is used, that is, *T*_1_ and *T*_2_. The threshold processing can be regarded as the test of function *T*, see (1) for details.

(1) $$\begin{array}{c} T=T\left[x,y,p\left(x,y\right),f\left(x,y\right)\right]. \end{array}$$

In (1), *T* represents the threshold, (*x*, *y*) represents a point in the image, *f*(*x*, *y*) represents the gray level corresponding to the point, and *p*(*x*, *y*) represents its local properties. If the point is taken as the center to obtain the average gray level of the neighborhood, the image after threshold processing can be defined as given in the following equation:

(2) $$\begin{array}{c} g\left(x,y\right)=\left\{\begin{array}{cc} 1, & f\left(x,y\right)>T,\\ 0, & f\left(x,y\right)\leq T. \end{array}\right.. \end{array}$$

In equation (2), *g*(*x*, *y*) represents an image after threshold processing. According to equation (2), the pixels marked 1 and 0 correspond to the target object and the background, respectively. After the binarization of the image is completed, the region can be repaired and merged by morphological operation. The most commonly used operations of region repair are image expansion and image corrosion. The former mainly refers to expanding the boundary points of binary objects and integrating the background points in contact with them so as to achieve the expansion effect of image expansion to the outside. This operation method is usually applied to filling the holes after image segmentation as shown in the following formula:

(3) $$\begin{array}{c} S=A⊕B=\left\{z\;|\;{\left(\hat{B}\right)}_{z}\cap A\neq \emptyset \right\}. \end{array}$$

*S* represents the expansion result of the binary image set; *B* represents the structural element used for expansion, and its value is 0 or 1. Equation (3) shows that the *S* is obtained by using the graph *B* to expand the graph *A*. The process diagram of expansion treatment is shown in Figure 2.

Figure 2(a) shows a simple graph set *A*; Figure 2(b) shows the structural element *B* and its image, which have a symmetrical and equal relationship with respect to the central point; Figure 2(c) shows the *S* obtained after *A* expansion, from which the expansion range can be clearly seen. Another operation of region repair is image corrosion. The action mechanism of this method is quite different from image expansion. Its principle is to eliminate the boundary points of objects and shrink them inward. It is usually applied to the separate processing of two connected objects. Image expansion and image corrosion are both effective ways to trim the target object. After local or overall processing, the corresponding change characteristics can be obtained. In order to maintain the main features and shape of the head contour, it is usually necessary to be careful when selecting structural elements and avoid being too large or too small. After the binary processing and morphological processing of the image, the target image will form multiple subregions, which need to be segmented and extracted by region growth algorithm so as to obtain the initial contour of the head. The last step of CT image segmentation technology is to construct the contour model, and the most common method is to construct the set active contour model through the level set method. Different from other solving methods of geometric curve evolution, the level set method does not directly track the motion of evolution curve but uses implicit expression to describe the plane closed curve. First, let the mathematical expression of the plane active curve be as given in the following equation:

(4) $$\begin{array}{c} C\left(p,t\right)=\left(x\left(p,t\right),y\left(p,t\right)\right). \end{array}$$

In equation (4), *p* represents any parametric variable and *t* represents time variable, then the evolution process of curve *C* in the direction of unit normal vector $\vec{N}$ is shown in the following equation:

(5) $$\begin{array}{c} \frac{\partial C}{\partial t}=V\left(C\right)\vec{N}. \end{array}$$

The curve evolution in equation (5) mainly includes two different forms of constant evolution and curvature evolution. In (5), it represents a velocity function that determines the velocity of each point on the active curve. The evolution of curves mainly includes two different forms of constant evolution and curvature evolution. The difference between them lies in the setting of velocity function, i.e., constant and curvature. The evolution of the former can be expressed as a partial differential equation shown in the following equation:

(6) $$\begin{array}{c} \frac{\partial C}{\partial t}=V_{0}\vec{N}. \end{array}$$

The evolution process of the latter is shown in the following formula:

(7) $$\begin{array}{c} \frac{\partial C}{\partial t}=ak\vec{N}. \end{array}$$

In equation (7), *a* represents a positive constant, and *k* can accurately describe the bending degree of the curve. Then, the level set equation is constructed, and the level set function *ψ* is defined as hypersurface. Its expression is shown in the following equation:

(8) $$\begin{array}{c} \psi \left(x\left(t\right),t=0\right)=\pm d. \end{array}$$

In equation (8), ±*d* represents the symbolic distance between point *x* and surface *C*_0_. If *x* is located inside the surface, take a negative value; otherwise, take a positive value with derivative *t*, then equation (9) can be obtained.

(9) $$\begin{array}{c} \psi_{t}+\sum_{i=1}^{N}\psi_{X_{i}}X_{t_{i}}=0. \end{array}$$

When it is in the vertical state, there is the following equation:

(10) $$\begin{array}{c} \sum_{i=1}^{N}\psi_{X_{i}}X_{t_{i}}=\left(\psi_{X_{1}}\cdots \psi_{X_{N}}\right)\left(\psi_{1_{t}}\cdots \psi_{N_{t}}\right)=F\left(x\left(t\right)\right)\left|\nabla \psi \right|. \end{array}$$

After evolution, the level set equation can be rewritten as in the following equation:

(11) $$\begin{array}{c} \psi_{t}+F\left|\nabla \psi \right|\approx 0. \end{array}$$

In equation (11), *ψ* represents the level set function, then the contour curve of the target can be expressed as in the following equation:

(12) $$\begin{array}{c} \gamma \left(t\right)=\left(x\;|\;\psi \left(x,t\right)=0\right). \end{array}$$

### 3.2. 3D Reconstruction Technology Based on Contour Extraction and Sampling

Three-dimensional reconstruction technology is an important research direction of scientific visualization. This technology can process the two-dimensional pictures obtained by medical imaging equipment and then obtain the three-dimensional model of corresponding organs and tissues. Three-dimensional reconstruction technology mainly includes three different types, namely, surface rendering, volume rendering, and digital geometric processing, among which surface rendering has the best application effect. There is a triangulation method based on surface contour in surface rendering, which mainly uses the small plane with the shape of triangle or polygon to place it in the boundary contour line as a filler to form a complete and smooth object surface. Firstly, two feature point sets *P* and *Q* are set, which are expressed as (13) and (14), respectively.

(13) $$\begin{array}{c} P=\left\{p_{i}\;|\;0\leq i\leq m\right\}. \end{array}$$

In (13), the value of *m* is greater than or equal to 3, and *p*_*m*_=*p*_0_.

(14) $$\begin{array}{c} Q=\left\{q_{i}|0\leq j\leq n\right\}. \end{array}$$

The value of *n* is also not less than 3, and *q*_*m*_=*q*_0_. *P* and *Q* are arranged in clockwise order in adjacent layers. Between the two, the three-dimensional reconstruction of the surface is completed by using triangulation. The applied triangle must meet four conditions at least one vertex *P* and one vertex *Q* in the triangle. If the intersection line between different triangles is not *P*_*i*_*Q*_*j*_ such an edge, it must not intersect. Any intersecting edge *P*_*i*_*Q*_*j*_ only belongs to two triangles that maintain adjacent relationship. Any point of a fault segment belongs to one of the adjacent triangles. A triangle meeting the four conditions can be called an acceptable surface as shown in Figure 3.

As can be seen from Figure 3, the two feature point sets are distributed up and down, and *P* and *Q* are the upper point set and the lower point set, respectively. Since the visible area of the triangle is small and contains a large number of triangular meshes, it needs to consume a lot of system resources every time rendering, so it is necessary to simplify the triangular mesh effectively. The simplified processing method mainly includes two types—point deletion and edge shrinkage. Its operation flow is shown in Figure 4.

Figure 4(a) shows the three basic steps of point deletion. First, select a point in the triangular mesh model to delete, then delete the edge with the target point as the vertex, and finally, all the holes are processed to obtain a new triangular mesh.  Figure 4(b) shows the operation steps of edge contraction, which is mainly to move and merge the two endpoints located on the same edge to make it a point so that the original edge changes its connected endpoint and moves to the new vertex. In contrast, the operation of edge shrinkage is more convenient. It can complete the processing of two endpoints at one time and obtain a better simplification effect. Therefore, the application scope of edge shrinkage is far greater than that of point deletion.

There is a lot of data redundancy in the image and video data collected by widely deployed cameras. In video surveillance data, a large number of images and video data have time, space, and statistical redundancy. In order to reduce redundant data and shorten image processing time, contour sampling will be carried out using curve data compression algorithm (Douglas–Peucker, DP). The algorithm is a global sampling algorithm, which can obtain ideal and accurate sampling results based on vector or area offset.

The geometric principle of contour sampling by the DP algorithm is shown in Figure 5.

It can be seen from Figure 5 that during the sampling process of the DP algorithm, any arc of all curves in the polygon contour can realize the approximation with arbitrary accuracy, and the accuracy of the approximation can be described objectively and accurately according to the maximum distance between the point on the arc and the upper chord of the arc. The irregular polygon contour in Figure 5 is defined as *V*, and *V*=〈*v*_0_, *v*_1_ … *v*_*n*_〉. Let *v*_*p*_ represent any vertex in *V*, then its distance from any straight line $\bar{v_{0}v_{n}}$ can be expressed as $d\left(v_{p},\bar{v_{0}v_{n}}\right)$, and the corresponding approximation error is shown in the following equation:

(15) $$\begin{array}{c} \delta_{DP}\left(\bar{v_{0}v_{n}},V\right)=\max\left(d\left(v_{p},\bar{v_{0}v_{n}}\right)\right)v_{p}\in V. \end{array}$$

In equation (15), *δ*_*DP*_ represents the approximation error, and then, a distance threshold *ε* used to represent the approximation accuracy is set. For all vertices in *V*, the distance between them and $\bar{v_{0}v_{n}}$ is calculated and compared one by one, and then, the vertex with the maximum distance is obtained, which is recorded as *v*_*p*1_. If the corresponding maximum distance $d\left(v_{p1},\bar{v_{0}v_{n}}\right)$ is less than the established threshold, it can be determined that the irregular polygon *V* can be replaced by the straight line $\bar{v_{0}v_{n}}$, which marks the end of the decomposition. If not, it is necessary to decompose the subcontour recursively until the conditions are met.

## 4. Experimental Design and Analysis

### 4.1. Edge Extraction Results and Contour Model of CT Image Segmentation Technology

Compared with the traditional image segmentation technology, CT image segmentation technology based on human anatomy is more effective and can obtain excellent segmentation effect when the target object has a large contrast with the background. This method adopts the unitary global threshold segmentation technology to easily realize the effective extraction and segmentation of image edges in the process of pixel-by-pixel scanning and marking. See Figure 6 for details.

Figures 6(a) and 6(b) are the original CT images of the head when the fault sequence is 20 and 40, respectively. After using the CT image segmentation technology based on human anatomy, the fault segmentation results of Figures 6(c) and 6(d) are successfully obtained, which correspond to two original images, respectively. It can be seen that the CT image segmentation technology based on human anatomy can obtain the more essential morphology and features of the target image and realize the significant improvement of image quality. In order to further explore the application effect of CT image segmentation technology, study and set different thresholds and analyze the gray histogram under different fault numbers, in order to obtain the effectiveness of CT image segmentation technology in distinguishing the target image from the background. The results are shown in Figure 7.

According to Figure 7, under the influence of different thresholds, there are some differences in the distribution of threshold histogram, but the overall difference is small, which shows that CT image segmentation technology has significant universality and efficiency and can realize the effective segmentation of target image and background without the interference of different thresholds. There is a close relationship between the extraction of the contour of the target image and the acquisition of the contour model. The higher the accuracy of the extraction of the former, the higher the quality of the latter. See Figure 8 for the convergence contour generated by different algorithms in approximation processing.

Figures 8(a)–8(c) are the approximation results of the traditional image segmentation technology. The difference lies in the number of iterations, which are 20, 40, and 60 in turn. The blue line represents the original contour of the target image, and the red line represents the approximate contour. According to Figures 8(a)to 8(c), with the increasing number of iterations, the similarity between the approximate contour and the original image shows a certain improvement, but there are still large differences between them. Figures 8(d)–8(f) show the approximation results of CT image segmentation technology based on human anatomy, and the iteration times are also 20, 40, and 60, respectively. By comparing and analyzing Figures 8(d)–8(f), it can be seen that there is no significant difference in the convergence contour generated under different iteration times, which is almost consistent, and the convergence contour is highly consistent with the original contour.

### 4.2. Surface Rendering and 3D Display Results

Set the layer spacing and point spacing between data to 3 mm and 0.418 mm, respectively, so that the data scale is 512 × 512 × 69. Subsequently, the experimental results of surface rendering are obtained as shown in Figure 9.

Figures 9(a) and 9(c) are the surface drawing results before fitting, and Figures 9(b) and 9(d) are the surface drawing results after fitting. Compared with the rendering results before and after fitting, the head CT scanning image after fitting is clearer and the reconstruction effect is better. Comparing the fitting effects under different threshold levels, it can be seen that when the threshold level is low, the 3D reconstruction effect is better. If the threshold is too large, a large number of scattered fragments will appear in the 3D reconstruction results. In order to further explore the impact of threshold on 3D reconstruction results, this study conducted 3D reconstruction experiments with different thresholds, recorded the time required for each experiment, and scored the 3D reconstruction results. See Table 1 for the results.

According to Table 1, with the increase in threshold, the time required for 3D reconstruction gradually decreases, indicating that the reconstruction efficiency shows an obvious improvement trend. Because a large number of discrete fragments will be displayed in the reconstruction results, the CT image of the head cannot be completely presented. Therefore, with the improvement of threshold and efficiency, the score of 3D reconstruction effect continues to decline.

## 5. Conclusion

At present, various diseases occur frequently in the medical community, and people's health is endangered by various diseases, among which head diseases are the most dangerous. It is very important to make effective diagnosis and treatment. In order to improve the level of medical diagnosis, this study will explore the mechanism of head CT image segmentation and three-dimensional reconstruction technology based on human anatomy and adopt different morphological operation methods and other measures, such as image expansion, image corrosion, point deletion, and edge contraction, in order to optimize head CT image segmentation technology and three-dimensional reconstruction technology. The experimental results show that under the influence of different thresholds, there are some differences in the distribution of threshold histogram, but the overall difference is small, which shows that CT image segmentation technology can effectively segment the target image and background. As for the three-dimensional imaging results themselves, the threshold has a great influence. The threshold is negatively correlated with the three-dimensional imaging time and the score of three-dimensional reconstruction results. This shows that in order to obtain better 3D reconstruction effect, it is necessary to ensure that the threshold is at a low level under the condition of reasonable time. The application effect of CT image segmentation technology and three-dimensional imaging technology based on human anatomy is good, which can provide reliable support for medical diagnosis and treatment.

## Figures and Tables

**Figure 1:** Different types of threshold histograms. (a) Single-threshold histogram; (b) multithreshold histogram.

**Figure 2:** Schematic diagram of image expansion process. (a) Graph set A; (b) structure element *B* and its image; (c) *S* obtained after expansion treatment.

**Figure 3:** Structural diagram of basic triangle.

**Figure 4:** Schematic diagram of simplified processing operation of triangular mesh. (a) Operation flow of point deletion; (b) operation flow of edge contraction.

**Figure 5:** Geometric principle of DP algorithm.

**Figure 6:** Extraction and segmentation results of head CT under different fault sequences. (a) CT image sequence tomography 20; (b) CT image sequence tomography 40; (c) fault 20 segmentation results; (d) fault 40 segmentation results.

**Figure 7:** Histogram distribution of head CT under different fault sequences. (a) Histogram distribution of fault 20; (b) histogram distribution of fault 40.

**Figure 8:** Comparison of approximation experimental results of two algorithms. (a) Traditional approximation results (20 iterations); (b) traditional approximation results (40 iterations); (c) traditional approximation results (60 iterations); (d) improved approximation results (20 iterations); (e) improved approximation results (20 iterations); (f) improved approximation results (20 iterations).

**Figure 9:** Comparison of surface fitting under different isosurfaces. (a) Draw the result before fitting when the threshold is small; (b) draw the result after fitting when the threshold is small; (c) draw the results before fitting when the threshold is large; (d) draw the result after fitting when the threshold is large.

**Table 1:** Effects of different thresholds on 3D reconstruction time and effect.

Threshold	Reconstruction time (s)	3D reconstruction effect score
5	42.75	93.47
10	41.04	89.58
15	36.57	84.52
20	33.25	82.09
25	31.33	79.63
30	26.42	76.88
35	22.85	71.64
40	19.13	66.25
45	15.57	59.87
50	12.47	51.26

## Data Availability

The data used to support the findings of this study are available from the corresponding author upon request.
